# The Imaging Diagnosis of Patients with Shoulder Pain Caused by Sports Injury

**DOI:** 10.1155/2022/5272446

**Published:** 2022-04-21

**Authors:** Xiaoqi Dong, Lu Wang

**Affiliations:** Sports Department, Harbin Institute of Technology, Harbin, 150001 Heilongjiang, China

## Abstract

The shoulder joint is the most complex and movable joint of the human body. A variety of diseases can affect the shoulder joint and cause shoulder pain. Sports injuries are an important and common cause of shoulder pain. In the clinical diagnosis of shoulder joint injury, the most commonly used diagnostic methods are X-ray photography and CT imaging, but X-ray photography has poor ability to distinguish shoulder joints and other tiny tissue structures and has a sense of inspiration for shoulder joint injuries. In addition, CT arthrography has a certain risk to the lesion and is easy to form trauma, and it cannot clearly show the shoulder joint structures such as the rotator cuff and the labrum. Therefore, this article conducts MR imaging diagnostic research on patients with shoulder pain caused by sports injuries and plays an important role in imaging. This article deeply studied the clinical manifestations of shoulder joint pain and image processing technology, designed a research experiment on imaging diagnosis results of patients with shoulder joint pain caused by sports injuries, selected 87 patients with shoulder joint pain in a hospital, and analyzed X-ray photography, CT imaging, and MR imaging diagnosis, three methods to compare the diagnostic accuracy and inspection results and conduct an in-depth analysis of the causes of shoulder joint injury. The experimental results showed that there were 87 patients with shoulder joint pain, 65 patients with rotator cuff tear were diagnosed using arthroscopy, and 63 patients with rotator cuff tear were diagnosed by MR imaging. The accuracy rate was as high as 95.6%. Among them, the proportion caused by sports injuries is the highest, reaching 56%.

## 1. Introduction

Shoulder joint injuries are easily affected by age, stress, and psychological trauma. Clinically, the main symptoms of shoulder joint trauma are shoulder joint pain, restriction of shoulder joint mobility, and decreased muscle strength. Because of the complex structure and shape of the shoulder joint, the injury of the shoulder joint has a great influence on the range of motion of the upper limbs. There is a need to further improve the diagnosis and treatment of joint injuries and improve the prognosis of patients.

MRI has gradually become one of the typical contents of clinical diagnosis and joint disease diagnosis. It plays an important role in the diagnosis and treatment of acute and chronic shoulder joint injuries and provides basic effects for the diagnosis and treatment of shoulder joint injuries. If the shoulder is injured, a torn rotator cuff is the most common clinical symptom. It is mainly a laceration of the supraspinatus tendon, which is divided into two types: complete tear and partial tear.

Nabhan et al. describe the incidence of injuries and illnesses during the 2014 Youth Olympic Games (YOG) in the United States during the Youth Olympic Games (YOG). There are methods of a retrospective analysis of the electronic health records of registered athletes at the American Youth Olympic Games (YOG). Medical malpractice refers to all medical services provided by medical service providers, including assessment, treatment, and prevention services. All medical conditions are classified according to the International Olympic Committee's injury report. The results of team USA consisted of 48 male athletes and 46 female athletes, aged between 14 and 18 years old, representing 20 sports. Among the 94 registered athletes, 54 athletes have a total of 346 medical visits, and each athlete has 3.7 medical visits. A total of 40 cases of injuries (14 cases of time-loss injuries, 26 cases of non-time-loss injuries) and 20 cases of diseases were recorded. This is equivalent to 43% of athletes injured, 21% of athletes sick, 426 injured, and 213 sick per 1,000 registered athletes. The most common body part for time-loss injuries is the knee (21%). It can be seen that the proportion of sports injuries is relatively high [1]. The rapid development of Park et al.'s liver imaging has improved the evaluation of the occurrence and development of liver cancer and the early diagnosis and treatment of liver cancer. In this case, discovering the development of early liver cancer is of great significance for improving patient survival and optimizing treatment strategies. Since early HCC is considered a precursor of progressive HCC, it is very important to accurately distinguish dysplastic nodules (DN), especially the difference between high-grade DN and early HCC. In clinical practice, these nodules are often referred to as “boundary liver nodules.” Summary: They discussed the imaging and pathological features of these boundary liver nodules and focused on the imaging changes during the progression of DN and early HCC, to gain an understanding of the occurrence and development of multistep liver cancer. Contrast-enhanced ultrasound, CT, and MRI combined with extracellular contrast agents are still a challenge for the detection and accurate diagnosis of liver junctional nodules. However, gadolinic acid-enhanced MRI may help improve the diagnosis of these borderline nodules. Key message: due to the net effect of incomplete angiogenesis and reduced portal blood flow in the early stages of liver cancer, borderline liver nodules usually appear as isovascular or hypovascular. Therefore, the precise identification of these nodules remains a challenging problem. In MRI using hepatobiliary contrast agents, the signal intensity of HCCs in the hepatobiliary phase (HBP) is considered a potential imaging marker. Hepatic junctional nodules appear as nonvascular and low-signal nodules on HBP, which are of great significance for predicting tumor behavior and determining appropriate treatment strategies. However, this is the application research of imaging in the field of liver [2]. In Bcker et al.'s background, in recent years, aerial sports have become more and more popular. As athletes take more and more risks to experience this adventurous spirit, the number of accidents has skyrocketed. The objective is to investigate the various injuries in airborne sports accidents, as well as the acute treatments these patients received and the first-level trauma center before and after admission. Methods: we have a major first-level trauma center in Switzerland for 235 hospitalized due to air sports injuries between 2010 and 2017. A retrospective chart analysis was performed on two patients, patient demographic data, injury patterns, emergency primary care procedures, and hospital care records. Results: in total, 718 of the 235 patients were injured; the spine was the most common site of injury, with 46.5% of the 143 patients injured (*n* = 334/718). 69 (15.5%) patients (nonspine) had chest involvement, followed by injuries of the lower and upper limbs, pelvis, head/face, and abdomen [3].

The innovations of this article are as follows: (1) combining qualitative research with quantitative research, fully combining research data with practical application value, and showing the practical value of this research; (2) combining theoretical research with empirical research, in-depth study based on the theoretical basis of imaging technology, combined with the actual situation of bone and joint clinical research for empirical investigation. This paper provides a development suggestion for the medical industry under the imaging theory and can also provide new ideas for the research on the diagnosis and treatment of shoulder joint injuries.

## 2. Research Methods of Imaging Diagnosis Results of Patients with Shoulder Pain Caused by Sports Injuries

### 2.1. Tendon and Muscle Disease

1. Tendon calcification

The clinical manifestations of shoulder tendon calcification can be asymptomatic, severe pain, or varying degrees of chronic pain, and pain can lead to a reduction in the range of movement of the shoulder joint [4]. Shoulder tendon calcification is common in middle-aged people. All tendons of the rotator cuff can be affected, and the suprasmus tendons are most often involved. Rotator cuff tendon calcification X-ray showed oval calcifications near the greater humerus tubercle, and MRI showed low signal nodules in the corresponding tendon.

(2) Tendon tear

The rotator cuff is composed of the tendons of the supraspinalis, subspinalis, teres minor, and subscapularis. It is a one-cuff-like structure covering the glenohumeral joint capsule, which supports and stabilizes the glenohumeral joint during shoulder joint movement. Role [5]: trauma, degeneration, and chronic injury can cause rotator cuff tears. Rotator cuff tears often involve the suprasuma tendon, and the tearing site is usually near the attachment site of the tendon. The long head of the biceps brachii tendon is in the shoulder joint, and the injury may also cause pain in the shoulder joint. MRI is the most suitable imaging method for the diagnosis of tendon rupture, with high sensitivity and specificity. Partial cracks appear as high signal areas of MRI tendons, and complete cracks appear as tendon ruptures and signal enhancement [6].

### 2.2. Labrum Disease

The glenoid labrum of the shoulder joint is a fibrocartilage structure attached to the circumference of the glenoid cleft and plays a role in strengthening the shoulder joint [7]. Labrum lesions include degeneration and tearing, which can cause shoulder joint pain. Labrum tears include petal tears, longitudinal tears, and anteroposterior tears of the upper labrum. Although labrum tears can occur alone, it is common clinically that the labrum is avulsed from the glenoid and the joint capsule tears. The glenohumeral joint is unstable. MRI is the best imaging method for the diagnosis of labrum tears. In addition to conventional scans, MRI shoulder arthrography and shoulder abduction and external rotation are required to detect some lesions. According to the extent of involvement and the way of tearing, labrum tears can be divided into many forms.

1. Bankart lesions: divided into cartilage and osteochondral lesions. Cartilage Bankart lesions refer to the avulsion of the anterior inferior labrum with the lifting and tearing of the adjacent glenoid periosteum; the osteochondral Bankart lesions are based on cartilage accompanied by a fracture of the anterior and lower edge of the glenoid
2. Anterior inferior labrum lesions with damage to the hyaline cartilage on the articular surface of the glenoid: mostly due to forced abduction, and most patients have pain in the front of the shoulder joint. This lesion is clearly shown under MRI shoulder arthrography
3. Sleeve avulsion of the anterior glenoid periosteum: it is also a variant of Bankart's disease, which is a complete avulsion and displacement of the anterior inferior labrum. The glenoid periosteum is lifted up but still connected with the glenoid. It is common after traumatic shoulder dislocation, which often leads to shoulder joint instability
4. Slap tear: refers to the anterior and posterior tear of the superior labrum, manifested as pain in the front of the shoulder joint. The disease is more common in athletes who make repeated throwing movements or others who repeatedly stretch the biceps labrum complex. It is divided into four types: type I is slight degeneration and surface wear; type II is a classic type, which represents the tear and separation of the superior labrum from the glenoid; type II is a barrel-shaped tear of the superior labrum; type IV is a tear of the superior labrum. The fissure separates and extends to the attachment site or tendon of the long head of the biceps brachii [8, 9].

Figure 1 shows the main manifestations of shoulder joint injuries.

### 2.3. Image Processing Technology Algorithm

After receiving the spiral CT scan, the patients in the research team need to undergo an image examination, send the relevant two-dimensional images to the base station, and perform image processing procedures. First, in order to prevent the scanned frame from participating in image reconstruction, the area needs to be adjusted [10, 11]. Next, construct MPR based on the observation and understanding of the bone window and soft tissue window, remove the tissues that affect the observation, expose the observation area, observe the patient's fracture displacement and fracture line direction, adjust the brightness and contrast appropriately, and save the relevant images. By adjusting the transparency of soft tissue, air, and fat, a satisfactory image is finally obtained [12, 13].

The basic functions of reading, displaying, and saving images are realized by calling OpenCV [14–16]. The image consists of a table. The black and white image is a one-dimensional two-dimensional matrix such as a chess board. The size of each point on the chessboard represents the gray level of the image unit. Depending on the image unit, a black and white image is formed. The color image is a three-dimensional table composed of three channels. Color images can be distinguished by b, g, r=cv2. Splitting can be achieved by splitting or separating channels [17]. In the case of a composite color image of 3 channels, you can call cv2.merge ([b, g, r]) to perform channel merging. The essence of digital image processing is grayscale processing. The formula for converting color pixels to grayscale pixels is applicable to OpenCV, and the formula is as follows:

(1) $$\begin{array}{c} \text{gray}=\left(0.14\;0.587\;0.299\right)\begin{array}{c} \text{B},\\ \text{G},\\ \text{R}. \end{array} \end{array}$$

The geometric transformation of the image requires two independent algorithms to complete the chapter of the geometric transformation of the image. First, convert the coordinates to pixel positions, and then, convert them to pixel positions. Second, it needs to be involved. The algorithm ends the gray value output of each pixel of the image.

The translation formula is:

(2) $$\begin{array}{c} \left(\begin{array}{c} \tilde{x}\\ \tilde{y}\\ 1 \end{array}\right)=\left(\begin{array}{ccc} 1 & 0 & t_{x}\\ 0 & 1 & t_{y}\\ 0 & 0 & 1 \end{array}\right)\left(\begin{array}{c} x\\ y\\ 1 \end{array}\right). \end{array}$$

*Tx* > 0 means moving along the *x*-axis square, and vice versa.

Scaling formula:

(3) $$\begin{array}{c} \left(\begin{array}{c} \tilde{x}\\ \tilde{y}\\ 1 \end{array}\right)=\left(\begin{array}{ccc} s_{x} & 0 & 0\\ 0 & s_{x} & 0\\ 0 & 0 & 1 \end{array}\right)\left(\begin{array}{c} x\\ y\\ 1 \end{array}\right). \end{array}$$

*S*_*x*_ > 1 means to zoom in in the horizontal direction and vice versa; *S*_*y*_ > 1means to zoom in the picture in the vertical direction, and vice versa.

Rotation formula:

(4) $$\begin{array}{c} \left(\begin{array}{c} \tilde{x}\\ \tilde{y}\\ 1 \end{array}\right)=\left(\begin{array}{ccc} \cos\alpha & \sin\alpha & 0\\ -\sin\alpha & \cos\alpha & 0\\ 0 & 0 & 1 \end{array}\right). \end{array}$$

When *a* > 0, turn clockwise to the right; otherwise, counterclockwise. This is achieved by calling cv2.rotate. Image rotation, scaling, etc. are collectively referred to as affine transformation.

Bilinear interpolation: the converted pixel *f*(*i* + *u*, *j* + *v*) is determined by the value of about 4 pixels (*i*, *j*), (*i* + 1, *j*), (*i*, *j* + 1), (*i* + 1, *j* + 1) corresponding to the original image coordinates.

(5) $$\begin{array}{c} f\left(i+u,j+v\right)=\left(1-u\right)\left(1-v\right)f\left(i,j\right),u\left(1-v\right)\left(i+1,j\right),\left(1-u\right)v\left(i,j+1\right),uv\left(i+1,j+1\right). \end{array}$$

In the above formula, *u* = |*i* − [*i*]|, *v* = |*j* − [*j*]|, (*i*, *j*) is the horizontal and vertical distance from the integer coordinates of the bell.

Increasing the contrast can solve the problem of low contrast caused by small image gray. Its purpose is to extend the gray level of the output image to a defined level so that the details of the image look more beautiful. Generally used are linear transformation, histogram normalization, gamma transformation, global uniform histogram, etc. [18].

Linear transformation:

(6) $$\begin{array}{c} O\left(r,c\right)=a*I\left(r,c\right)+b. \end{array}$$

In the formula, the range of *r* and *c* is 0 < *I* = (*r*, *c*) ≤ 255; in the case of *a* > 1, the contrast of the output image will increase, 0 < *a* < 1, the contrast of the output image will hardly decrease. When *b* > 0, the brightness increases. Otherwise, the brightness will decrease. The bisecting linear transformation is to perform different linear transformations on different pixel width values. In other words, it 0 < *I* = (*r*, *c*) ≤ 255 is divided into multiple*O*(*r*, *c*) = *a*∗*I*(*r*, *c*) + *b*, and multiple matching items are used to achieve linear conversion.

Normalization of the histogram:

(7) $$\begin{array}{c} O\left(r,c\right)=\frac{O_{\max}-O_{\min}}{I_{\max}-I_{\min}}\left(I\left(r,c\right)-I_{\min}\right)+O_{\min}. \end{array}$$

In formula (7), *I*(*r*, *c*) represents the input image, and *I*_max_, *I*_min_represents the max and Min of the image gray level.

Global histogram equalization:

(8) $$\begin{array}{c} q\approx \frac{\sum_{k=0}^{p}{\text{hist}}_{I}\left(k\right)}{H*W}*256-1, \end{array}$$

(9) $$\begin{array}{c} O\left(r,c\right)=\frac{\sum_{k=0}^{I\left(r.c\right)}{\text{hist}}_{I}\left(k\right)}{H*W}*256-1. \end{array}$$

hist_*I*_(*k*) represents the number of pixels whose gray value is equal to *k*, where *k* ∈ [0,255]. Global histogram equalization steps: first, calculate the gray histogram of the image; calculate the gray histogram cluster histogram, the relationship between a gray histogram. Finally, according to the gray-scale mapping relationship obtained in the third step, the gray-scale value of each pixel of the output image is obtained cyclically [19].

### 2.4. MRI Chemical Shift Imaging Technology

The imaging technology of chemical magnetic shift imaging is also called phase imaging and inverse phase imaging. Chemical shift imaging technology is based on the chemical effects of proton transfer on fat and water molecules [20, 21]. At present, most clinical shift imaging technologies use the corrected GREET1 WID sequence that can easily receive reverse phase and phase images. Currently, the segmented GREET1 WI sequence is used for new MRIs over 1.5 T. The dual-sound technology can simultaneously shoot in-phase images in the same direction during the same scanning process, and the obtained images can be compared.

At present, chemical shift imaging technology is widely used clinically. The phase diagram is ordinary T1WI. Before introducing the clinical application of chemical shift imaging, we must first understand the characteristics of inverse phase imaging. The inverse phase image has the following main characteristics [22, 23].

The signal of mixed adipose tissue is significantly weakened, and its weakening degree generally exceeds the signal of selective fat saturation technology. 30% of the special tissue signal comes from lipids, and 70% comes from water molecules. When the selective saturation method is used to suppress fat, even if all lipid signals are completely suppressed, 70% of the characteristics of water molecules will not change. In other words, the attenuation amplitude of the signal is 30%. In the inverted image, not only 30% of the lipid signal disappears, but 70% of the water molecule signal is also compensated by 30% of the primary fat. The organization only maintains 40% of the original signal, and the attenuation amplitude of the signal reaches 60%.

The traces of net adipose tissue should not be significantly weakened. In tissues close to pure fat, such as subcutaneous fat, midgut fat, and perfume, the signal source is mainly fat, which contains almost no water molecules. Since the transverse magnetic medium where the two protons cancel each other is small, the tissue signal will not be greatly reduced.

In the inverted image, a black line representing the outline of the organ will be displayed at one end of the surrounding organs with rich adipose tissue. The general organ signal mainly comes from water molecules, and the surrounding adipose tissue signal mainly comes from fat. Therefore, in the inverted image, the environment of the marked body and adipose tissue will not drop significantly, but both organs have organs (water molecules). Moreover, fat is on the boundary of each wax at the same time, the signal is obviously reduced to the inverted image, and acne appears.

The current clinical application of chemical shift imaging technology and the clinical application of chemical change imaging technology are mainly applied to abdominal organs. The main uses are as follows: (1) diagnosis of adrenaline working diseases. Adrenal tumors contain more lipids, so the signal intensity of backlit images usually drops significantly. The sensitivity of chemical shift imaging in judging whether adrenaline clusters are adenomas increased from 70% to 80%, and the specificity increased from 90% to 95%; (2) diagnosis and differential diagnosis of fatty liver: the fat in the liver is higher than normal; (3) others: the application of chemical shift imaging technology is also helpful for the diagnosis and identification of vascular fat in the kidney or liver muscle [24].

## 3. Experiment on Imaging Diagnosis Results of Patients with Shoulder Joint Pain Caused by Sports Injury

1. Selection of research objects for imaging diagnosis of patients with shoulder joint pain caused by sports injuries

In this article, 87 patients with shoulder joint injuries who were hospitalized from May 2017 to May 2018 were selected. The clinical data of all patients are complete, with clinical symptoms of shoulder joint injury; they provided the information and agreed. They were randomly divided into the previous X-ray group, spiral CT group, and MRI diagnosis group, with 28 cases, 28 cases, and 31 cases, respectively. The age of these patients was 17-60 years old, with an average age of 22.3 ± 3.2 years old. Injuries included rotator cuff tear, labrum injury, and supraspinatus tendon tear. All injuries were caused by sports injuries. There was no significant difference in general information between the 3 groups of patients (*P* > 0.05), and they were comparable.

(2) Research methods of imaging diagnosis in patients with shoulder pain caused by sports injuries

This article mainly uses Philips 3.0 MRI to examine the patient, selects a special scanning system for the limbs and joints, and assists the patient to adopt a supine position, keep the upper limbs in a neutral position, and use a coil to wrap the shoulder joint of the patient's side; give the disease Patients with oblique coronal position PDWIFSET1WI, horizontal axis position PDWIFSET1WI, oblique sagittal position PDWI fat suppression sequence scan, PDWI-FST2WI if necessary, parameter setting: layer thickness 3.0 mm~4.0 mm, matrix 288 × 224, FOV is 18 × 18 mm. Arthroscopy: the patient sits on the beach or in a chair, is anesthetized regularly, and uses traditional medicine to help diagnose the shoulder joint by applying the assault joint system [25].

The position of the shoulder scanner and the patient: ACHEVIA 1.5 T magnetic coordinate scanner with 8-channel coil is dedicated for shoulder joints. The patient is in a lower position with the upper limbs placed on both sides of the body, and the scan is performed regularly in a neutral position (the thumb is rotated upward or slightly outward). In order to make patients feel comfortable and reduce mobility, a thin foam pad is placed on the elbow. The patient first undergoes regular MRI examinations using the following parameters [26]. Tendinitis on the shoulder is also suspected to be abnormal. The following is the method.

MRI scan sequence and parameters of the shoulder joint: routine MRI scans of the shoulder joint include sequences: fast spin echo TIYJI-weighted imaging (TSET1wITR/TE = 45O/15 ms), fast spin echo T2), J1-weighted imaging (TsET2wITR/TE = 4000/80 ms), fast spin echo T2-weighted fat pressure image (T2WISPAIR, TR/TE = 4000/30 ms). Scanning field of view (field of view, FOV) 160 mm × 160 mm, image acquisition matrix and display matrix 256 × 56, scanning layer 3 mm, and layer spacing 0.3 mm [27].

Magnetic scanning method: previous shoulder MRI scans include CT scan, external coronary artery, and external oval level. All patients underwent TSSET2 WI + FS scans and were placed on the images scanned for horizontal and horizontal scan scans. The horizontal installation lines (TSSET1 WI, TSSET2 WI, and TSSET2 WI + FS) are parallel to the upper arm tendons. The front end of the scanning range must be from the subhead and back to the subframe. The scan line outside the ellipse (TSSET2 WI + Fs) is perpendicular to the outer side of the coronary artery. In other words, the scan line is perpendicular to the upper spinal cord. Swing from the scapula to the largest vertebra of the wrist without losing the outer layer including the upper and lower spines [28].

MR shoulder arthrography examination method. The patient underwent shoulder arthrography immediately or within 7 days after the routine MRI examination. Contrast agent: dilute 0.5 ml Gd-DTPA into 100 ml normal saline, and extract 10-15 m12~5 m15% lidocaine for contrast.

Specify the lower end of the puncture point (3 points). After disinfection, insert the needle vertically, and the layer becomes transparent during the needle insertion process, and the resistance and hardness of the puncture point and the upper boundary can be felt. The measured penetration depth has now been reached. Ask the assistant to hold the patient's upper arm and slowly tighten it to internally rotate it while inserting a 0.5-1.0 needle. Before you feel the sense of loss, take out the resistant syringe and continue to improve the contrast by 12-15 ml if the contrast coefficient is damaged, no resistance or low resistance. Contrast scan within 40 minutes after the completion of the injection include transection, oblique coronal position, oblique sagittal fat pressure, and oblique coronal no compression JIlT1 weighted image (TSE, TR/TE = 450/15 ms, F0V = 160 mm). All MR images were analyzed blindly by two deputy chief physicians of the bone group. All patients use shoulder arthroscopy as the “gold standard” to calculate its sensitivity and accuracy [29, 30].

(3) Observation index of imaging diagnosis of patients with shoulder joint pain caused by sports injury

Analyze the image data of MR1 and MR1 of the shoulder joint to clarify the structure of the bone (including the classification of limb morphology, the changes of brain tumors, and the formation of bone bud cells), the structure of the rotating cuff (including the changes in signal and rotating morphology), the subcutaneous, the flow of body fluids, and the state of the lower lip (including signal changes, spectral shape, and obvious high-signal labrum tear).

## 4. Statistical Methods

Using the software SPSS20.0, the count data of the shoulder joint injuries of the three groups of patients were represented by the rate (%), using the *χ*^2^ test and the exact probability method, and the test standard *a* = 0.05.

## 5. Performance in Imaging

### 5.1. MR Imaging Manifestations of Rotator Cuff Tear

Rotator cuff tear is mainly the tear of the supraspinatus tendon. According to the degree of tear, it can be divided into partial tear and complete tear. External coronary artery scans have the highest analysis of MRI images with rotating cuffs and local fissures. This is mainly manifested in T2WI and STIR sequences, as well as tendon injury accompanied by abnormal signals at the injury site such as the continuity of the tendon. The MR image of a total laceration showed that the local tendon alignment was interrupted, and the T2 WI or STIR alignment signal penetrated the entire tendon.

### 5.2. MR Imaging Manifestations of Labrum Injury

Labrum tears are often accompanied by joint oozing. On the MR display, there is a high signal representation similar to the T2 WI or STIR sequence lips, which can include the surface of the pronunciation, which can extend the limit or the basis of the laboratory. The height signal 2 extending from the lips to the labrum is known.

### 5.3. Normal Imaging Manifestations of the Shoulder Joint

The general magnetic resonance imaging performance of the shoulder joint is as follows. The cross-section and oblique axis of the shoulder joint are in the best configuration. The muscles of the abdomen show the average signal, the tendons show the low signal, and the upper and lower parts of the spinal cord show the average signal. For patients with shoulder joint injuries, rotating cuffs and breast injuries are the most important symptom forms of hypofunction of the shoulder joint.  Figure 2 is a flow chart of imaging diagnostic experiments for patients with shoulder joint pain caused by sports injuries.

## 6. Imaging Diagnosis Results of Patients with Shoulder Pain Caused by Sports Injuries

### 6.1. Comparative Analysis of Imaging Diagnosis Results of Patients with Shoulder Joint Pain

The clinically commonly used inspection methods for shoulder joint injury mainly include CT arthrography, X-ray photography, and other inspection methods, but X-ray films cannot accurately distinguish the microstructure of the shoulder joint, and its specificity in the diagnosis of shoulder joint injury. And the sensitivity is not high; CT imaging will cause certain trauma to the damaged part of the shoulder joint, and the damage to the labrum, rotator cuff, and other tissue structures of the shoulder joint cannot be effectively presented, and with the continuous development of clinical medical technology, the effectiveness of MR inspection methods in the diagnosis of shoulder joint injuries has received widespread attention, and MR images have three-dimensional multiplanar imaging functions, which can effectively distinguish the soft tissues of the shoulder joints with high resolution. At the same time, MR images have the advantages of nonradioactive, noninvasive, and better tissue control comparability which have been widely used in clinical practice.

Table 1 shows the comparison table of the number of people detected and the number of missed people who were examined by the three methods. Among them, there were 28 patients in the X-ray group, 22 of which were detected, and 6 were missed; of the 28 patients in the CT group, 25 were detected, and 3 were missed; 31 were detected by MR imaging, and 6 were missed. In 0 cases, the detection rate was 100%.

As can be seen from Figure 3, the detection rate of the MR imaging group was significantly higher than that of the other two groups (*P* < 0.05), showing a certain advantage.

Table 2 shows the comparison table of the detection rate and missed detection rate of the three methods for patient inspection. The detection rate of X-ray photography was 82.3%, and the missed detection rate was 17.7%; the detection rate of CT arthrography was 95.6%, and the missed detection rate was 4.4%. The detection rate of MR imaging diagnosis group was 100%, and the missed detection rate was 100%. 0%.

It can be seen from Figure 4 that MR imaging has the highest detection rate and the lowest missed detection rate, indicating that MR imaging is the most effective for the diagnosis of bone and joint injuries, and the detection rate is much higher than the other two traditional methods. It helps doctors diagnose and treat bone and joint injuries and improve the efficiency of diagnosis.

Table 3 shows the X-ray method, CT method, and MR method. The imaging method diagnoses the three angles and adds the arthroscopic diagnosis as the most accurate comparison of the diagnosis results.

It can be seen from Figure 5 that there are 87 patients with shoulder joint pain in this article, 65 patients with rotator cuff tear were diagnosed using arthroscopy, and 63 patients with rotator cuff tear were diagnosed by MR imaging, with an accuracy rate of 95.6%; using arthroscopy, 14 cases of labrum injury were diagnosed, and 13 cases were diagnosed by MR imaging. Compared with the diagnosis results of arthroscopy, the MR imaging group is closest to the diagnosis results of arthroscopy, with an accuracy rate of 95.6%. The diagnosis results of X-ray and CT groups are not much different, but they are far lower than the diagnosis results of arthroscopy.

It can be seen from Table 4 that the result of MR imaging diagnosis of rotator cuff tear is as high as 96%, which is infinitely close to the diagnosis of arthroscopy; the diagnosis of labrum injury with X-ray diagnosis is poor, and the diagnosis rate is only 58%. The diagnosis rate of supraspinatus tendon tear using MR imaging reached 100%.

It can be clearly seen from Figure 6 that MRI is a good indicator of shoulder joint injury and also has a good effect on symptoms such as cuff rotation and breast injury. The diagnosis rate of shoulder injuries is high.

Labrum injury is another common form of shoulder joint injury, and its state is more complicated. All fatal injuries are shown on local joints. The overall crack shows a high signal on the tendon surface, extending to the fat line under the defatted muscle. Moreover, MRI can not only quickly diagnose shoulder joint injuries but also has a more sensitive diagnostic function for nontraumatic shoulder joint injuries. The shoulder joints can also be enlarged. The characteristic signal can make a correct judgment.

### 6.2. Comparison of Inspection Effects and Accuracy of Shoulder Joint Injury Diagnosis Methods

Table 5 and Figure 7 show the comparison of the inspection effects of the three methods. It can be seen from the table that the total effective rate of MR imaging diagnosis is 98%, the total effective rate of X-ray diagnosis is 64%, and the total effective rate of CT diagnosis is 83%. MR imaging diagnosis results are significantly higher than the other two diagnosis methods, and its clinical value is the highest.

It can be seen from Table 6 that in terms of the diagnostic accuracy rate, the total number of patients in this experiment is 87, the MR imaging diagnostic accuracy is 78 cases, the diagnostic accuracy rate reaches 90%, and the diagnostic accuracy rate is as high as 98%, statistically significant (*χ*^2^ = 4.234, *P* < 0.05).

The shoulder joint is the most complicated joint in the human body, usually composed of 3 bones (clavicle, shoulder joint, wrist) and 4 joints (scapula joint, sternum joint, their connection is composed of muscles, tendons, and ligaments). The 4 shoulder joints move at the same time to ensure smooth upper limb movement.

There are many reasons for shoulder joint injuries, such as shoulder pain caused by age, sports, trauma, and other diseases. From the comparison of the causes and effects of shoulder joint injuries in Table 7 and Figure 8, it can be seen that sports injuries account for the highest proportion of shoulder joint injuries, reaching 56%, followed by traffic accidents, reaching 47%. Therefore, when using the shoulder joints daily, pay attention to the strength and strength, especially for athletes who need to repeat overhead movements.

## 7. Conclusions

This article focuses on the imaging diagnosis results of patients with shoulder joint pain caused by sports injuries. Three methods of X-ray photography, CT imaging, and MR imaging are used to diagnose rotator cuff tear, labrum injury, and supraspinatus tendon tear. Diagnosis and analysis and comparison of the accuracy of the diagnosis results through arthroscopy showed that the imaging diagnosis results of patients with shoulder joint pain are highly accurate. In addition, the causes of shoulder joint injuries were analyzed to avoid shoulder joint injuries from the source.

The innovations of this article are as follows: first, the combination of qualitative research and quantitative research, fully combining research data with practical application value, and showing the practical value of the research in this article; second, the combination of theoretical research and empirical research, in-depth study based on the theoretical basis of imaging technology, combined with the actual situation of bone and joint clinical research for empirical investigation.

This article still has some shortcomings: although the MR imaging diagnosis method used in this article has high inspection accuracy, the equipment and inspection costs are expensive, which limits its popularity and application to a certain extent; the second is that the equipment scan time is long. It may be unbearable for patients; thirdly, patients who have metal implants or metal foreign bodies in their bodies cannot use it. There are certain requirements for patients. However, with the development of the times and economy, MR imaging diagnosis will be more adapted to the pace of the times, and further improvements will be made to make the popularization and application scope wider. In the future work, we will study appropriate medical diagnosis methods and means from more perspectives based on the existing technology and level and continuously improve the quality of medical diagnosis and treatment.

## Figures and Tables

**Figure 1:** Main manifestations of shoulder joint injury.

**Figure 2:** Flow chart of imaging diagnosis test for patients with shoulder pain caused by sports injury.

**Figure 3:** Detection of shoulder joint injuries in three groups of patients.

**Figure 4:** The proportion of shoulder joint injuries detected in the three groups.

**Figure 5:** Comparison of the number of patients diagnosed.

**Figure 6:** The proportion of shoulder joint diagnosed by three methods.

**Figure 7:** Comparison of three inspection methods.

**Figure 8:** Comparison of the causes of shoulder joint injury.

**Table 1:** Detection of shoulder joint injuries in three groups of patients.

Group	*N*	Number of people checked out	Number of missed diagnosis
Conventional X-ray film group	28	22	6
Spiral CT group	28	25	3
MR imaging examination group	31	31	0
*χ* ^2^	—	11.14	12.38
*P*	—	<0.05	<0.05

**Table 2:** The proportion of shoulder joint injuries detected in the three groups.

Group	*N*	The detection rate (%)	Missed diagnosis rate (%)
Conventional X-ray film group	28	82.3	17.7
Spiral CT group	28	95.6	4.4
MR imaging examination group	31	100.00	0

**Table 3:** Diagnosis of shoulder joint injury by three methods.

Group	*N*	Rotator cuff tear	Labrum injury	Supraspinatus tendon tear	Accuracy rate/%
Conventional X-ray film group	87	56	8	2	78.9
Spiral CT group	87	58	9	3	80.2
MR imaging examination group	87	63	13	8	95.6
Arthroscopy	87	65	14	8	100.00

**Table 4:** The proportion of shoulder joint diagnosed by three methods.

Group	Rotator cuff tear/%	Labrum injury/%	Supraspinatus tendon tear/%
Conventional X-ray film group	0.86	0.58	0.25
Spiral CT group	0.89	0.64	0.375
MR imaging examination group	0.96	0.93	1
Arthroscopy	1	1	1

**Table 5:** Comparison of three inspection methods.

Inspection method	*N*	The effect is better	The effect is average	The effect is poor	Total effective rate
X-ray examination	87	12 (0.14)	56 (0.64)	19 (0.22)	56 (0.64)
Spiral CT examination	87	36 (0.42)	45 (0.52)	6 (0.06)	72 (0.83)
MR imaging	87	58 (0.67)	28 (0.32)	1 (0.01)	85 (0.98)
*χ* ^2^	—	—			5.121
*P*	—	—			0.024

**Table 6:** Comparison of diagnostic accuracy of three methods.

Inspection method	*N*	The accuracy is high	Average accuracy	The accuracy is poor	Diagnostic accuracy
X-ray examination	87	56 (0.64)	15 (0.17)	16 (0.18)	68 (0.78)
Spiral CT examination	87	65 (0.75)	13 (0.15)	9 (0.10)	78 (0.90)
MR imaging	87	78 (0.90)	9 (0.10)	0 (0)	85 (0.98)
*χ* ^2^	—	—			4.234
*P*	—	—			0.039

**Table 7:** Comparison of the causes of shoulder joint injury.

	Sports injury/%	Traffic accident/%	Bodybuilding/%	Other/%
Rotator cuff tear	56	47	35	22
Labrum injury	23	15	21	19
Rupture of supraspinatus tendon	32	12	42	13

## Data Availability

The data that support the findings of this study are available from the corresponding author upon reasonable request.
